The article "Nanocurcumin Prevents Hypoxia Induced Stress in Primary Human Ventricular Cardiomyocytes by Maintaining Mitochondrial Homeostasis" was retracted in 2025. Reasons: errors in the data; errors in the images; duplicated images; duplicated data.

# Nanocurcumin Prevents Hypoxia Induced Stress in Primary Human Ventricular Cardiomyocytes by Maintaining Mitochondrial Homeostasis

**DOI:** 10.1371/journal.pone.0139121

**Published:** 2015-09-25

**Authors:** Sarita Nehra, Varun Bhardwaj, Lilly Ganju, Deepika Saraswat

**Affiliations:** Experimental Biology Division, Department of Experimental Biology, Defence Institute of Physiology and Allied Science, Defence Research and Development Organization, Timarpur, New Delhi, India; University of Pecs Medical School, HUNGARY

## Abstract

Hypoxia induced oxidative stress incurs pathophysiological changes in hypertrophied cardiomyocytes by promoting translocation of p53 to mitochondria. Here, we investigate the cardio-protective efficacy of nanocurcumin in protecting primary human ventricular cardiomyocytes (HVCM) from hypoxia induced damages. Hypoxia induced hypertrophy was confirmed by FITC-phenylalanine uptake assay, atrial natriuretic factor (ANF) levels and cell size measurements. Hypoxia induced translocation of p53 was investigated by using mitochondrial membrane permeability transition pore blocker cyclosporin A (blocks entry of p53 to mitochondria) and confirmed by western blot and immunofluorescence. Mitochondrial damage in hypertrophied HVCM cells was evaluated by analysing bio-energetic, anti-oxidant and metabolic function and substrate switching form lipids to glucose. Nanocurcumin prevented translocation of p53 to mitochondria by stabilizing mitochondrial membrane potential and de-stressed hypertrophied HVCM cells by significant restoration in lactate, acetyl-coenzyme A, pyruvate and glucose content along with lactate dehydrogenase (LDH) and 5' adenosine monophosphate-activated protein kinase (AMPKα) activity. Significant restoration in glucose and modulation of GLUT-1 and GLUT-4 levels confirmed that nanocurcumin mediated prevention of substrate switching. Nanocurcumin prevented of mitochondrial stress as confirmed by c-fos/c-jun/p53 signalling. The data indicates decrease in p-300 histone acetyl transferase (HAT) mediated histone acetylation and GATA-4 activation as pharmacological targets of nanocurcumin in preventing hypoxia induced hypertrophy. The study provides an insight into propitious therapeutic effects of nanocurcumin in cardio-protection and usability in clinical applications.

## Introduction

Cardiomyocyte hypertrophy appears as an adaptive process under hypoxia in order to meet the increased oxygen demand and maintain homeostasis, however prolonged oxidative stress might induce (patho-) physiological events [1,2]. Histone acetylation remains a key regulators for induction of cardiomyocyte hypertrophy [3]. Histone acetylation by p-300 HAT promotes transcription of the DNA and activates hypertrophic gene expression [4]. In contrast, histone deacetylase (HDAC) prevents acetylation of histones and thus down-regulates gene expression [4]. Studies have shown that increased p-300 HAT activity induces cardiac hypertrophy both *in vitro* and *in vivo* [5,6]. But whether of hypoxia promotes p-300 HAT activity in cardiomyocytes remains un-elucidated. Although hypertrophy remains an acclimatizing strategy of cardiomyocytes under hypoxia, sustained oxidative stress is known to induce cytological damages at least in part, by activating cascade of stress-responsive events including mitochondrial damage, redox imbalance and apoptotic cell death [7–12]. Hypoxia induced cardiomyocyte damage is inevitably associated with disruption of mitochondrial function and induction of programmed cell death or apoptosis [13,14]. An otherwise rare phenomenon in terminally differentiated cardiomyocytes, apoptosis might possess serious health hazards and may lead to life-threatening clinical situations and requires attention [15,16]. Since preservation of mitochondrial function is critical to cardiac performance, it is important to assess the changes in mitochondrial homeostasis under stress [17].

The tumour suppressor p53 plays central role in maintaining cell-viability, cell-cycle regulation and apoptosis. The p53 undergoes MDM2 (Murine double minute 2) mediated degradation [18] and remains inactive by binding to c-Jun NH_2_-terminal kinase (JNK)[19] and accumulation of free p53 is not observed in the cytoplasm or cellular compartments under normal conditions. However stress-induced functional modification and stabilization promote p53 accumulation by preventing its ubiquitin mediated degradation and promotes dissociation from JNK-p53 complex [20]. Accumulation of active p53 plays a crucial role in mediating free radical associated DNA-damage and mitochondrial dysfunction. Hypoxia induced oxidative stress has been shown to accumulate p53 in oxygen-sensitive cardiomyocyte [21–23]. Oxidative stress thus promotes compartmentalization and trafficking of a fraction of total cellular p53 towards mitochondria prior to nucleus and initiates cellular apoptotic events by promoting oxidative damage, disrupting mitochondrial outer-membrane potential (ΔΨ_m_), activating caspases and promoting cell cycle arrest [24,25]. This chain of signalling events eventually leading to apoptosis is induced by excessive ROS leakage from the mitochondrial electron transport chain (*e*.*t*.*c*.) and disrupts MnSOD activity. Since ROS remains important regulator of p53 induced cellular damage, it is of prime importance to investigate the impact of excessive ROS leakage on (patho-) physiology of cardiomyocytes [26]. Depending upon the severity of hypoxic stress, active p53 may lead to cell-cycle arrest in actively proliferating cells or initiate apoptotic cell death in post-mitotic cells [27,28]. Since hypoxic stress promotes compromise in mitochondrial function and p53 has been known to incur mitochondria mediated pathological damages, it remains important to assess whether hypoxia induced translocation of p53 to mitochondria exerts damaging cellular events in hypertrophied cardiomyocytes.

Use of anti-oxidant therapies emerges out as an important countermeasure to protect from hypoxia induced damages. Natural dietary curry spice, curcumin has been known as pharmacological countermeasure that rescues the cells from stress-induced damages [29,30]. But low biological stability and poor bio-availability make it unsuitable to be used as a therapeutic agent. However, use of nanocurcumin complexes has been explored in a number of studies for improving bio-stability and bio-availability of curcumin to improve pharmacological properties of curcumin [31–33]. In this regard, we have shown the cardio-protective efficacy of nanocurcumin in rodent embryonic H9c2 cells under hypoxia [34]. However, in order to establish a better causal relationship between hypoxia induced cardio-damages in humans with in vitro experimentations, improvement is required in in vitro studies by using appropriate cell lines. Here, we used terminally differentiated post-mitotic adult human ventricular cardiomyocytes (HVCM) as in vitro model of hypoxia induced hypertrophy since these cells reflect a closer biological association to cardiac-pathologies in humans and better disclose the cellular signalling behind to these pathologies due to intrinsic mechanisms [35].

Thus, in the present study, we investigated whether hypoxia induces pathological damages in hypertrophied HVCM cells under hypoxia and assessed the modulatory role of p53 in same. Here we show tremendous cardio-protective efficacy of nanocurcumin in HVCM cells experiencing severe mitochondrial stress due to modulation of critical cellular signalling cascades.

## Materials and Methods

### Experimental design

Experiments were designed to cover two main aspects of the study, i.e. evaluation of efficacy of nanocurcumin in ameliorating hypoxia induced hypertrophy and damage in HVCM cells and analysis of changes in hypoxia induced translocation of p53 to mitochondria and associated defects in mitochondrial function under hypoxia. All experiments were compared to raw curcumin as control.

The cells were grown in 6, 12 or 96 well plates (Nunc, Denmark) with a cell count of 10^4^−10^5^ viable cells/cm^2^. The HVCM cells were incubated in the CO_2_ incubator (Galaxy 170R, New Burnswick) and maintained at 37°C temperature and 5% CO_2_ overnight for adhesion. The cells were grown to 70–80% confluence before onset of experiments. The one set of confluent cells were subjected to normoxia i.e. 21% O_2_ and another set with 0.5% O_2_ i.e. hypoxia condition (0.5% O_2,_ 5% CO_2,_ 94.5% N_2_) in the incubator. The cells were divided into six groups, i.e. normoxia only (N), normoxia plus curcumin (N+C), normoxia plus nanocurcumin (N+NC), hypoxia only (H), hypoxia plus curcumin (N+C) and hypoxia plus nanocurcumin (H+NC) for experiments. Stock solutions of curcumin or nanocurcumin were prepared in neutral PBS (Phosphate buffered saline)(1mg/ml) by sonication for 15 minutes at 4°C (pulse cycle 9s, amplitude 40%)(SONICS VIBRA CELL, Sonic and Materials Inc.) as previously described [36,37]. Stock solutions were diluted at concentrations of 100 to 1000 ng/ml in neutral PBS) as vehicle for assessment of improvement in cellular viability at 24 h of hypoxia. Cells were subjected to different durations of hypoxia, i.e. for 1, 3, 6, 12 and 24 h to study time course of p53 mediated imbalance in cellular redox status and onset of mitochondrial damage. The anti-hypertrophic efficacy of nanocurcumin was assessed by estimating changes in p-300 HAT and HDAC activities and confirmed by GATA-4 expression levels [38]. The cellular signalling from promoting survival under stress was assessed by studying p53-JNK signalling pathway.

### HVCM cells

Adult human primary ventricular cardiomyocytes were procured from PromoCell^®^ GmbH (C12810), Heidelberg, Germany and maintained in myocyte growth medium (PromoCell^®^ GmbH, C22070). Molecular grade chemicals for cell-culture were procured from SIGMA ALDRICH or otherwise stated. Nanocurcumin of ultra-pure quality, was obtained as a kind gift from Prof. Santosh Kar (KIIT University, India) [39]. Native curcumin (C7727) was purchased from SIGMA ALDRICH.

### Isolation of cellular fractions and protein estimation

Cultured cells were de-adhered using trypsin-EDTA (0.1% v/v) for 5–10 minutes and counted by using Neubauer haemocytometer. Cells were homogenized on ice in RIPA (Radio-immunoprecipitation) buffer composition included Tris-HCl 50 mM, NaCl 150 mM, SDS 0.1%, NP-40 1%, Deoxycholate 0.5% and protease inhibitor cocktail (PIC)(MP Biomedicals, LLC, France) (1μl/mL buffer), centrifuged at 8000 rpm for 10 minutes and the supernatant containing cytosolic fraction was collected immediately on ice. To isolate mitochondrial fractions, the pellet was dissolved in mitochondrial isolation buffer (Mannitol 250 mM, HEPES 5 mM, 0.5 mM EGTA) and centrifuged at 25000 rpm for 30 minutes to isolate clear supernatant containing mitochondrial fractions as described previously [40]. To isolate nuclear fraction, the pellet was re-dissolved in nuclear protein isolation buffer (20 mM HEPES, 420 mM NaCl, 1.5 mM MgCl_2_, 0.2 mM EDTA, 0.5 mM DTT, 0.5 mM PMSF, 0.1% PIC) on ice for 20 minutes and centrifuged at 12000 rpm for 30 minutes. The supernatant containing clear nuclear fraction was collected. The protein estimation was done with Lowry’s method using bovine serum albumin (BSA) as internal standard [41]. The cytosolic, mitochondrial and nuclear extracts of the cells were stored at -80°C until further use.

### Assessment of hypoxia induced hypertrophy and apoptosis

Hypoxia induced apoptosis was assessed in HVCM cells by neutral red (E895, AMRESCO) uptake assay [42] and further confirmed by evaluation of caspase-3,-7 release as cellular markers of apoptosis by fluorescence activated cell sorting (FACS) using commercially available kit (APT403, Calbiochem, Millipore) and performed according to manufacturer’s instructions. Cardiomyocyte hypertrophy was assessed by evaluating levels of atrial natriuretic factor (ANF) using ELISA kit (EIA05048R) according to manufacturer’s instructions and increment in FITC-phenylalanine (NNPN-2, Millipore) uptake assay according to method described by Hebert *et*. *al*. as hallmark markers of hypertrophy and increment in protein synthesis respectively [43]. The enhancement in amino acid uptake was represented as percentage change in amino acid uptake by cardiomyocytes under hypoxia. Hypertrophied cells were also visualized by fluorescent microscope after staining with Alexa fluor 488-phalloidin (A12379, Molecular Probes) for assessment of cell size.

### Evaluation of p-300 HAT and HDAC activity

Histone acetylation is a critical marker of cardiac hypertrophy [3]. Studies have shown that curcumin inhibits p-300 mediated HAT activity and blunts hypertrophy[38]. Thus, it remains important to assess whether hypoxic stress induces hypertrophy by affecting p-300 HAT activity in HVCM cells. The effect of nanocurcumin on p-300 HAT activity was assessed in nuclear fractions of cardiomyocytes using commercially available kit (SensoLyte® HAT (p300), AS-72172, AnaSpec Inc.) according to manufacturer’s instructions and represented as percentage change in p-300 HAT activity. Nuclear expression of p-300 was further confirmed by immunofluoresnce staining using rabbit polyclonal anti-p300 antibody (sc585, 1:100) and developed against alexa-fluor 597 (A-11012, 1:1000, Molecular Probes). The cells were counterstained with DAPI (4', 6-diamidino-2-phenylindole, D1306, Molecular Probes) and alexa-fluor 488 phalloidin (A12379, Molecular Probes) to visualize nuclei and cytoskeleton. The cells were immediately mounted (ProLong^®^ Gold Antifade Reagent, P36934, Molecular Probes) and visualized (100X) under high resolution fluorescent microscope (IMAGER.M2, AxioCam MRc5, Carl Zeiss). Hypoxia induced acetylation of histone 3 and 4 was further confirmed by western blot analysis. In order to check the effect of nanocurcumin on HDAC, the nuclear fractions were assessed for HDAC activity using commercially available kit (Cayman Chemicals, 10011563,) and expressed as percentage change in HDAC activity.

### Co-localization of p53 and mtHsp70 by immunofluorescence

Mitochondrial Hsp70 (mtHsp70) assists the translocation of p53 to mitochondrial under stress [44]. Thus, evaluation of mtHsp70 remains an important mitochondrial marker to be evaluated in order to identify p53 translocation to mitochondria. The evaluation of p53 trafficking to mitochondria in HVCM cells under hypoxia was done using co-immunofluorescence for p53 and mtHsp70. HVCM cells were incubated in blocking buffer (3% bovine serum albumin, BSA, in 0.1% triton-X 100) at room temperature for 1 h and then overnight at 4°C in rabbit polyclonal anti-p53 (sc6243, 1:50) and mouse monoclonal anti-mtHsp70 (MA3-028, ThermoFischer Scientific, 1:100) following two washes in PBS. The cells were then incubated with anti-rabbit cyanine-3 (1:2000, Molecular Probes) or anti-mouse-FITC (sc2855, 1:1000) at room temperature for 2 h and counterstained with 0.1% DAPI. The cells were immediately mounted and visualized under fluorescent microscope.

### Prevention of mitochondrial translocation of p53 in HVCM cells under hypoxia

In order to investigate whether hypoxia induced hypertrophy in HVCM cells and associated mitochondrial stress were dependent upon translocation of p53 to mitochondria; we assessed the ANF levels of HVCM cells by preventing entry of p53 to mitochondria. The cells were divided into five groups, i.e. normoxia (N), hypoxia (H), hypoxia+CsA (H+CsA), hypoxia+curcumin (H+C) and hypoxia+nanocurcumin (H+NC). To achieve the same, HVCM cells were treated with cyclosporin A (CsA) as blocker of p53 entry to mitochondria (1μM, 30024, SIGMA ALDRICH) as described previously [45]. Cells were treated with cyclosporin A before exposure to hypoxia and assessed for levels of p53 in mitochondria and ANF levels as marker of hypertrophy in HVCM cells and compared to normoxia and hypoxia controls.

### Evaluation of mitochondrial homeostasis

Mitochondrial homeostasis and function were assessed by evaluation of changes in metabolic, energetic and redox function under hypoxia in terms of change in acetyl coenzyme A (acetyl co-A) concentration, pyruvate concentration, glucose levels, lactate levels and lactate dehydrogenase (LDH) activity, ΔΨ_m_, efficiency to generate ATP and assessment of MnSOD activity using fluorescence microscopy, fluorescence-activated cell sorting (FACS) analysis and biochemical estimations.

Changes in acetyl co-A concentration (MAK039, SIGMA ALDRICH), pyruvate concentration (MAK071, SIGMA ALDRICH), glucose (Gluc-PAP, Randox), lactate concentrations (MAK064, SIGMA ALDRICH) and LDH activity (MAK066, SIGMA ALDRICH) were assessed using commercially available kits and performed according to manufacturer’s instructions. Further confirmation of mitochondrial metabolic and substrate switching from fatty acids to glucose was done by evaluation of GLUT-1 and GLUT-4 expression levels[46,47]. The ΔΨ_m_ were evaluated using rhodamine 123 (R8004, SIGMA ALDRICH) and counterstained by propidium iodide (P3566, Molecular Probes) by using FACS at different time points of 1, 3, 6, 12 and 24 h. Assessment of mitochondrial energetic efficacy was done by measurement of cellular ATP pool (A22066, Invitrogen) and confirmed by evaluating p-T172-5' adenosine monophosphate-activated protein kinase (AMPKα) activity (KHO0621, Invitrogen) using commercially available kits and performed according to manufacturer’s instructions. Qualitative assessment of MnSOD content was performed using commercially available kit (HCS232FR, Millipore) and performed according to manufacturer’s instructions. Quantitative assessment of MnSOD was done according to method described previously [40].

### Western Blot

For western blot analysis, 30 μg of cytosolic, nuclear or mitochondrial proteins were resolved in 10% or 15% SDS-PAGE (Sodium dodecyl sulphate-polyacrylamide gel electrophoresis). The resolved proteins were transferred on to nitrocellulose membrane (Millipore, USA) by semi-dry trans-blot system (BioRad, USA) at 15 V for 45 min. The membranes were blocked in blocking buffer (3% Bovine serum albumin in tris-buffered saline-Tween, 0.1%) for one hour at room temperature. The membranes were washed with TBST (0.1%) thrice at 10 minutes interval and then were incubated with rabbit polyclonal anti-p53 antibody (sc6243, 1:1000, SantaCruz Biotechnology, USA), rabbit polyclonal anti-c-Jun (sc44, 1:1000, SantaCruz Biotechnology, USA), rabbit polyclonal anti-c-Fos (sc52, 1:500, SantaCruz Biotechnology, USA), rabbit polyclonal anti-histone 3 (06–599, 1:500, Millipore), rabbit polyclonal anti-histone 4 (06–866,1:500, Millipore), rabbit polyclonal anti GLUT-4 (sc7938, 1:400, SantaCruz Biotechnology, USA), rabbit polyclonal anti GLUT-1(sc7903, 1:500, SantaCruz Biotechnology, USA), goat polyclonal anti GATA-4 (sc1237, 1:250, SantaCruz Biotechnology, USA) or rabbit polyclonal p-GATA-4 (sc32823, 1:250, SantaCruz Biotechnology, USA) antibodies for 2–3 h at room temperature. The membranes were again washed with TBST thrice at 10 minutes interval and re-incubated with bovine anti-rabbit-IgG-HRP (horse radish peroxidise) or mouse-anti-goat-IgG-HRP antibodies (1:25,000) (SantaCruz Biotechnology, USA) at room temperature for 2 h. The membranes were washed twice and visualized by using chemiluminescent substrate and captured the image (SIGMA ALDRICH, USA) on photographic film.

### Evaluation of oxidative stress under hypoxia

Hypoxia induced oxidative stress was evaluated using enzymatic and non-enzymatic cellular anti-oxidants i.e. free radical generation by ROS estimation, GSH/GSSH, lipid peroxidation and xanthine oxidase assays at different time points of 1, 3, 6, 12 and 24 h of hypoxia by quantitative methods.

Free radical generation was assessed by the method described by Cathcart *et*. *al*. [48]. Reduced glutathione (GSH) and oxidised glutathione (GSSG) levels in cytosolic fractions were determined fluorimetrically by the method of Hissin and Hilf [49]. Lipid peroxidation was measured in cellular cytosolic fraction in terms of formation of malondialdehyde as described by Utley *et*. *al*. [50]. To evaluate generation of superoxide radicals under hypoxia, assessment of xanthine oxidase activity was done in cytosolic fractions of HVCM cells using Xanthine Oxidase Fluorometric assay kit (Cayman Chemical, 10010895) according to manufacturer’s instructions.

### Statistical Analysis

Quantitative data was expressed as mean ± standard deviation (SD) for each experimental group. The results were analysed for statistical significance using one-way or two-way ANOVA. Differences were considered statistically significant at p≤0.05, p≤0.005, p≤0.01 and p≤0.001. Experiments were performed thrice (n = 3) for statistical significance.

## Results

### Nanocurcumin prevents hypoxia induced apoptosis

Hypoxia insult reduced the cellular viability to 21% (p≤0.01) when compared to normoxia control cells as depicted by neutral red uptake assay as observed in Fig 1A. Further, it was confirmed using caspase-3,-7 release assay by FACS that nanocurcumin treatment (500 ng/ml) significantly improved cellular viability under hypoxia (85.5%, p≤0.01) better than curcumin as depicted in Fig 1B. Since increment in nanocurcumin dose beyond 500ng/ml did not further improved cellular viability under hypoxia, the same dose was used for further experiments.

**Fig 1:** Nanocurcumin improves cellular viability under hypoxia: (A) Hypoxia insult caused decline in cell viability (20%) compared to normoxia control cells by 24 h. (B) Nanocurcumin treatment at 500 ng/ml significantly improved cellular viability (89%) by 24 h of hypoxia exposure and confirmed by FACS. Curcumin treatment did not show significant improvement in cellular viability at any time point. No significant change in cell viability was observed in nanocurcumin or curcumin treated cells under normoxia. Nanocurcumin treatment at 500 ng/ml was used for further experiments. Values are mean ± SD, significant values represented as ^@@^p≤0.01 *vs* normoxia and ^#^p≤0.01 *vs* hypoxia. Non-significant changes are designated as ns.

### Nanocurcumin prevents hypoxia induced hypertrophy

Hypoxia induced hypertrophy in HVCM cells which was assessed by increase in cell size, FITC-phenylalanine uptake assay and confirmed by changes ANF levels as shown in Fig 2. HVCM cells exposed to hypoxia showed increment in cell size by 18% (as shown in Fig 2B), increment in amino acid uptake by 73% and up-regulation of ANF levels by 2.9 times (as shown in Fig 2C) after 24 h of hypoxia exposure compared to normoxia control cells. Treatment of cardiomyocytes with nanocurcumin after 24 h of hypoxia reduced cell size by 38% (*vs* 26% in curcumin), amino acid uptake by 42.8% (*vs* 56.3% in curcumin) and ANF levels by 64% (*vs* 25% in curcumin)(as observed in Fig 2D) compared to cells exposed to hypoxia only. Better improvement in cellular viability and prevention from hypertrophy were thus evident in HVCM cells treated with nanocurcumin than curcumin under hypoxia. These findings suggest that nanocurcumin indeed prevents hypoxia stress in HVCM cells better than curcumin. However, changes in cellular viability and ANF levels were not observed in nanocurcumin or curcumin treated cells under normoxia.

**Fig 2:** Nanocurcumin prevents hypoxia induced hypertrophy in HVCM cells: (A, B) Fluorescent staining of HVCM cells (60X) with actin filaments (green) and nuclei (blue) under various experimental groups showed increase in cell size in hypoxia exposed cells compared to normoxia controls. (C) Increment in FITC-phenylalanine uptake was observed in cells exposed to hypoxia compared to normoxia control. (D) Increase in ANF levels were observed within 1 h of hypoxia and reached maximum by 24 h of hypoxia. Treatment with nanocurcumin significantly restored the cell size and FITC-phenylalanine uptake under hypoxia when compared to curcumin treated cells and cells exposed to hypoxia only. Nanocurcumin treated cells showed tremendous restoration in ANF levels under hypoxia at all the time points compared to curcumin treated cells. No significant changes in ANF levels, cell size or FITC-phenylalanine uptake was observed in cells exposed to normoxia after treatment with nanocurcumin or curcumin. Values are mean ± SD, significant values represented as ^@@^ p≤0.01 *vs* normoxia, *p≤0.05 *vs* hypoxia, ^#^p≤0.01 *vs* hypoxia, ^@^ p≤0.005 *vs* hypoxia and ^$ $^ p≤0.001 *vs* hypoxia. Bar represents 50 μm.

### Nanocurcumin prevents hypoxia induced hypertrophy by preventing p-300 HAT activity and GATA-4 levels

Histone acetylation, controlled by p-300 HAT and HDAC activities, is an important check point for induction of hypertrophy. Since maximum up-regulation of ANF was observed in cells exposed to 24 h of hypoxia, the p-300 HAT and HDAC activities were assessed in HVCM cells exposed to 24 h of hypoxia as shown in Fig 3A–3C. It was found that hypoxia insult increased p-300 HAT activity (63.34% *vs* normoxia control) in HVCM cells depicting induction of hypertrophy (S1 Fig). Also, to investigate the effect of nanocurcumin on hypo-acetylation activity, the HDAC activity was also assessed. Hypoxia insult decreased HDAC activity in HVCM cells (by 42.19% *vs* normoxia control) confirming that hypoxia induced hypertrophy in HVCM cells was dependent on histone acetylation activity. This was further confirmed by western blots of acetylated histone 3 and 4 as depicted in Fig 3B and S1 Fig. We further confirmed induction of hypertrophic genes in HVCM cells under hypoxia by checking the expression levels of GATA-4. It was found that phosphorylation and activation of GATA-4 was up-regulated in hypoxia exposed cells. Nanocurcumin treatment was found highly effective than curcumin in down-regulating p-GATA-4 expression in HVCM cells under hypoxia. This finding was corroborated with the observation that nanocurcumin treatment increased the HDAC activity in HVCM cells significantly (by 46% in nanocurcumin *vs* 9% in curcumin compared to hypoxia control). Nanocurcumin treated cells showed decrease in p-300 HAT activity under hypoxia (decreased by 52.14% *vs* 14% in curcumin) compared to hypoxia control cells. No change in p-300 HAT or HDAC activity was observed in nanocurcumin or curcumin treated cells under normoxia.

**Fig 3:** Effect of nanocurcumin on p-300 HAT and HDAC activities in HVCM cells under hypoxia: Histone acetylation by p-300 was up-regulated with a corresponding decline in HDAC activity in cardiomyocytes under hypoxia depicting that hypoxia induced hypertrophy dependent upon p-300 HAT and HDAC activity (A and C). Nanocurcumin treatment significantly down-regulated p-300 HAT and up-regulated HDAC activity in HVCM cells under hypoxia compared to cells exposed to hypoxia only. This was further confirmed by western blot analysis of GATA-4 and p-GATA-4 levels along with acetylated histone 3 and 4 (B). However, curcumin treatment did not prevent histone acetylation under hypoxia. Also, nanocurcumin or curcumin treated cells did not show change in p-300 HAT activity under normoxia. Values are mean ± SD, significant values represented as ^@@^ p≤0.01 *vs* normoxia, *p≤0.05 *vs* hypoxia and ^#^p≤0.01 *vs* hypoxia. Non-significant changes are depicted as ns. Scale bar represents 50μm.

### Hypoxia induced stress, but not hypertrophy, was dependent upon mitochondrial transition of p53

The damages observed in HVCM cells might be due to oxidative stress experienced by the cells. In order to recognize a causal relationship between hypoxia induced hypertrophy and damages experienced by HVCM cells, it was important to assess the effect of hypoxia on cardiomyocyte hypertrophy in absence of p53 translocation to mitochondria. To accomplish the same, we evaluated the extent of hypertrophy and mitochondrial homeostasis by preventing translocation of p53 to mitochondria by using CsA, a blocker of mitochondrial translocation of p53. The p53 levels and ANF expression levels were assessed in HVCM cells exposed to 24 h of hypoxia since maximum expression of these markers were observed in cells exposed to 24 h of hypoxia as shown in Fig 4A and 4B. It was found that CsA treatment effectively prevented translocation of p53 to mitochondria. However, preventing translocation of p53 to mitochondria had no effect on changes in ANF levels in HVCM cells under hypoxia as shown in S2 Fig. This depicts that induction of hypoxia induced hypertrophy in HVCM cells was independent of translocation of p53 to mitochondria. However, the mitochondrial stress experienced by hypertrophied HVCM cells was dependent upon translocation of p53 to mitochondria.

**Fig 4:** Hypoxia induced hypertrophy is independent of translocation of p53 to mitochondria: The dependency of translocation of p53 to mitochondria on induction of hypertrophy in HVCM cells under hypoxia was estimated by blocking entry of p53 to mitochondria by treatment with CsA. Treatment of HVCM cells with CsA prevented p53 translocation to mitochondria but did not affect ANF levels in HVC cells exposed to hypoxia for 24 h. However, treatment HVCM cells with nanocurcumin significantly reduced p53 translocation to mitochondria and down-regulated ANF levels. Values are mean ± SD, significant values represented as ^@@^p≤0.01 *vs* normoxia, ^#^p≤0.01 *vs* hypoxia, *p≤0.05 *vs* hypoxia.

### Time-course disruption of ΔΨ_m_ under hypoxia in HVCM

Maintenance of mitochondrial membrane potential is detrimental for sustaining normal physiological functioning of cells. The compromise in ΔΨ_m_ under hypoxia may result in cellular damaging events and lead to apoptosis. In order to assess the disturbance in ΔΨ_m_, we analysed the HVCM cells stained with ΔΨ_m_ sensitive dye and screened using FACS as shown in Fig 5A–5C and S3 Fig. It was found that ΔΨ_m_ was disturbed as early as 1 h of hypoxia which corroborated with the observation that MnSOD activity was down-regulated in HVCM cells by 1 h (decreased by 66%) of hypoxia compared to normoxia as observed in Fig 6A–6C and S4 and S5 Figs. This indicates that hypoxia elicits damage to oxygen-sensitive cardiomyocytes as early as 1 h of hypoxia exposure as depicted by disruption of ΔΨ_m_ and down-regulation of mitochondrial protective antioxidant mechanism. Maximum restoration in disruption of ΔΨ_m_ and restoration of MnSOD activity (decreased by 43% compared to normoxia) were observed in 24 h of hypoxia exposed HVCM cells as shown in Figs 5C and 6C. Also, nanocurcumin better restored the ΔΨ_m_ and MnSOD activity at all the time points than curcumin. No significant change was observed in HVCM cells treated with nanocurcumin or curcumin under normoxia.

**Fig 5:** Effect of nanocurcumin on ΔΨ_m_ in HVCM cells under hypoxia: (A) Hypoxia insult disrupted ΔΨ_m_ as early as 1 h of exposure caused in HVCM cells as depicted by FACS. (B) Curcumin treatment did not show any significant improvement in ΔΨ_m_ till 6 h of hypoxia and maximum protection was observed by 24 h of hypoxia. (C) Nanocurcumin treatment significantly restored the ΔΨ_m_ by 3 h of hypoxia than curcumin treated cells and maximum restoration was achieved by 24 h of hypoxia.

**Fig 6:** Nanocurcumin restored MnSOD levels cells under hypoxia: (A) MnSOD activity showed gradual decline with increment of duration of hypoxia as shown by fluorescent staining. (B) Curcumin treatment did not show significant restoration in MnSOD activity when compared to hypoxia control cells. (C) Treatment with nanocurcumin restored MnSOD activity in time dependent manner. Nanocurcumin significantly restored MnSOD activity in HVCM cells under hypoxia than curcumin treated cells under hypoxia when compared to cells exposed to hypoxia only. Random fields were captured by fluorescent microscope at 40 X magnification. At least 70 images were taken for each group and fluorescence intensity was quantized by using ImageJ software. Bar represents 10 μm.

### Nanocurcumin prevents translocation of p53 to mitochondria

The translocation of p53 to mitochondria is an initial event in the cascade that leads to cellular damaging events by disturbing mitochondrial homeostasis. We observed that p53 localization to mitochondria was increased under hypoxia within 1 h of exposure along with concomitant up-regulation of mtHsp70 as observed in Fig 7A and 7B. However, cytoplasmic levels of p53 and mtHSP70 increased upon hypoxia exposure as shown in Fig 7C. The channelization of p53 to mitochondria preceded the disruption of ΔΨ_m_ and down-regulation of MnSOD activity under hypoxia. This suggests that localization of p53 to mitochondria initiates damaging mitochondrial events which are accomplished in the form of down-regulation of protective anti-oxidant mechanisms and disruption of ΔΨ_m_ in HVCM cells under hypoxia. Treatment with nanocurcumin prevented translocation of p53 to mitochondria by down-regulating mtHsp70 levels and subsequent damage under hypoxia than curcumin as shown in Fig 7A–7C. Also, the up-stream targets of p53 activation, i.e. c-Fos and c-Jun were down-regulated in hypoxia exposed cells as observed in Fig 8A–8D. Nanocurcumin treatment effectively up-regulated c-Fos and c-Jun, thus down-regulating p53 induced cellular damage in HVCM cells under hypoxia as shown in Fig 8A–8D.

**Fig 7:** Nanocurcumin prevents hypoxia induced mitochondrial translocation of p53 in HVCM cells: Translocation of p53 in mitochondria (mito) in HVCM cells was time-dependent and initiated within1 h of hypoxia. Nanocurcumin prevented p53 translocation to mitochondria in HVCM cells under hypoxia better than curcumin (A, B). Also, enhancement in levels of p53 (Red) and mtHsp70 (Green) was observed after hypoxia insult in HVCM cells after 24 h (C). Nanocurcumin treatment down-regulated p53 and mtHsp70 levels better than curcumin treated cells under hypoxia. Bar represents 10 μm.

**Fig 8:** Nanocurcumin imparts cardio-protection in HVCM cells by activation of c-Jun/c-Fos: Hypoxia insult prevented c-Fos and c-Jun expression in HVCM cells upto 24 h of hypoxia and thus promoted translocation of p53 to mitochondria. Treatment of HVCM cells with nanocurcumin promoted c-Fos accumulation as early as 1 h of hypoxia and prevented p53 mediated cell-death whereas curcumin treated cells showed significant up-regulation of c-Fos and c-Jun by 6–12 h of treatment under hypoxia showing that nanocurcumin is frequently available to the cells compared to curcumin. Nanocurcumin treated cells showed higher expression of negative regulators of p53 accumulation, i.e. c-Jun and c-Fos in HVCM cells under hypoxia, depicting that improved bio-availability and stability of nanocurcumin prevents hypoxia induced damage in cardiomyocytes.

### Nanocurcumin preserved mitochondrial function under hypoxia

Oxidative stress elicits cellular demand of energy which is fulfilled by generation of more ATP by oxidative phosphorylation and simultaneously, carbohydrates are utilized as prime source of energy in-spite of lipids. In order to assess hypoxia induced changes in metabolic parameters in HVCM cells, we examined the changes in metabolic and bio-energetic function of mitochondria by evaluating acetyl co-A and pyruvate concentrations along with ATP levels and p-AMPKα activity. Also, the levels of lactate and glucose were evaluated to assess the effect of hypoxia on mitochondrial metabolism. We found that HVCM cells showed decrease in ATP, acetyl co-A and pyruvate concentrations and increase in p-AMPKα activity under hypoxia (0.5% O_2_, 24 h) as shown in Fig 9A and 9B. This was accompanied with increase in lactate concentration and LDH activity in HVCM cells as shown in Fig 9C. This was accompanied with increase in glucose uptake by HVCM cells depicting a possible shift in substrate specificity from lipids to carbohydrates under oxygen scarcity as observed in Fig 9D. To confirm the same, expression levels of GLUT-1and GLUT-4 were estimated. GLUT-1 and GLUT-4 are the foetal and adult isoforms of glucose transporter in myocardium respectively and are expressed in foetus and matured organisms [51]. However, stress-induced metabolic changes are associated with reversal of expression of these glucose transporters. Studies have well established that stress induced up-regulation of GLUT-1 and down-regulation of GLUT-4 in adult myocardium is associated with a metabolic substrate switch from lipids to carbohydrates[51,52]. In the present study, we found that hypoxia induced up-regulation of GLUT-1 and down-regulation of GLUT-4 which confirmed metabolic substrate switching in HVCM cells as shown in Fig 9E and 9F. These expression levels were significantly restored by nanocurcumin treatment in HVCM cells under hypoxia when compared to curcumin treated cells. The concomitant findings with up-regulation of glucose uptake in HVCM cells confirm that HVCM cells experienced a substrate switch from lipids to carbohydrates under hypoxia. This metabolic switch was well restored in nanocurcumin treatment under hypoxia compared to curcumin.

**Fig 9:** Nanocurcumin prevents hypoxia induced mitochondrial stress in HVCM cells: Hypoxia insult caused severe decline in ATP levels and increase in p-AMPKα activity (A) increase in acetyl co-A and pyruvate concentrations (B). Also, there was observed in increase in lactate content and LDH activity in HVCM cells (C) along with glucose uptake (D) in HVCM cells under hypoxia, depicting that hypoxia induced energy deficit in cardiomyocytes. This was further confirmed by western blots of GLUT-1 and GLU4 (E, F). Nanocurcumin treatment restored the cellular ATP levels and p-AMPKα activity by 24 h of hypoxia exposure to normal levels than curcumin treated cells when compared to cells exposed to hypoxia only. Nanocurcumin treated cells showed restoration in acetyl co-A and pyruvate concentrations, lactate content and LDH activity along with glucose uptake and expression levels of glucose transporters, whereas curcumin treated cells did not show significant restoration. Values are mean ± SD, significant values represented as ^@^p≤0.05 *vs* normoxia, ^@@^ p≤0.01 *vs* normoxia *p≤0.05 *vs* hypoxia and ^#^p≤0.01 *vs* hypoxia. Non-significant changes are designated as ns.

Under hypoxia, mitochondrial generation of ATP is decreased and levels of p-AMPKα increase to stimulate enhancement of ATP synthesis to maintain vital functions. However, prolonged oxidative stress induces down-regulation of p-AMPKα levels and ATP synthesis is compromised as observed in Fig 9A. Since maximum efficacy of nanocurcumin in restoration ΔΨ_m_ (82% compared to hypoxia only) and MnSOD (128% compared to hypoxia only) were observed in 24 h of hypoxia, we evaluated the efficacy of nanocurcumin in restoration of mitochondrial bio-energetic capacity after 24 h of hypoxia to HVCM cells. The efficacy of mitochondria to perform glycolysis was assessed by evaluating acetyl coenzyme A activity and pyruvate content as markers of oxidative stress induced metabolic changes. It was found that acetyl co-A concentration increased after 24 h of hypoxia with parallel decrease in pyruvate content and increase in lactate concentration (33.7% *vs* normoxia), glucose uptake (25.6%) and LDH activity (35.5% *vs* normoxia) depicting switching of substrate specificity from fatty acids to sugars to meet the enhanced energy requirements under hypoxia. Nanocurcumin treatment restored the acetyl co-A, pyruvate, lactate content and LDH activity in HVCM cells under hypoxia. However, curcumin did not show any significant result. Nanocurcumin treated cells showed significant restoration in acetyl co-A (48%), pyruvate (47%), glucose uptake (13.3%), lactate concentration (24%) and LDH activity (16%) compared to hypoxia control whereas curcumin treated cells did not show significant restoration. It was also found that ATP levels were halved and p-AMPKα activity increased (by 200%) under hypoxia compared to normoxia controls depicting energy deficit in cardiomyocytes as shown in Fig 9A. Treatment with nanocurcumin restored ATP levels (173%) and corresponding p-AMPKα activity (by 63%) in HVCM cells under hypoxia depicting maintenance of mitochondria bio-energetic function and homeostasis better than curcumin when compared to cells exposed to hypoxia only. Since mitochondrial complex V is involved in oxidative phosphorylation mediated ATP generation, these findings illustrate that nanocurcumin preserved mitochondrial function under hypoxia stress possibly by regulating complex V activity in HVCM cells.

### Nanocurcumin protects from hypoxia induced oxidative damage

Oxygen-sensitive cardiomyocytes experience severe oxidative stress under hypoxia. We analysed the effect of nanocurcumin in ameliorating cellular enzymatic and non-enzymatic antioxidants under hypoxia. Disturbance in GSH/GSSG content (decreased by 47%, as shown in Fig 10A) and increment in lipid peroxidation (3.9 times, as shown in Fig 10B) excessive ROS leakage (2.1 times, as shown in Fig 10C) along with changes in xanthine oxidase activity (1.7 times increase, as shown in Fig 10D) and MnSOD activity (0.38 times decline, as shown in Fig 10E) were observed under 24 h of hypoxia compared to normoxia control cells. The extent of oxidative damage corroborated with disruption to ΔΨ_m_ post translocation of p53 to mitochondria suggesting that p53 might affects cellular redox-machinery in order to maintain homeostasis. Nanocurcumin treatment was found to be highly significant in restoration of GSH/GSSG (129% *vs* 89% in curcumin, as shown in Fig 10A) reduction in lipid peroxidation (70% *vs* 32% in curcumin) as shown in Fig 10B and reduction in excessive ROS leakage (38% *vs* 11% in curcumin) as shown in Fig 10C including restoration in xanthine oxidase activity (32% *vs* 18% in curcumin) as observed in Fig 10D and MnSOD activity (14.5% *vs* 6.3% in curcumin, as observed in Fig 10E) in HVCM cells under hypoxia. No significant change in redox status was observed in nanocurcumin or curcumin treated cells under normoxia.

**Fig 10:** Nanocurcumin protects HVCM cells by restoring oxidative balance: Hypoxia stress disturbed cellular redox balance as depicted by increase in ROS leakage and lipid peroxidation and concomitant decrease in GSH/GSSG content, xanthine oxidase activity and MnSOD activity. Nanocurcumin treatment showed significant improvement in redox status when compared to curcumin treated cells under hypoxia and cells exposed to hypoxia only. No significant change in redox status was observed in cells treated with curcumin or nanocurcumin under normoxia. Values are mean ± SD, significant values represented as ^@^p≤0.05 *vs* normoxia, ^#^p≤0.01 *vs* hypoxia, *p≤0.05 *vs* hypoxia.

## Discussion

Oxidative stress induced hypertrophy and apoptosis remains a serious clinical situation in cardiac (patho-) physiology [14]. Accumulation of p53 plays a crucial role in oxygen-sensitive cardiomyocytes by modulating mitochondrial function. Recent findings have shown that hypoxia induced translocation of p53 to mitochondria elicits serious pathological injuries to cardiomyocytes which involves damage to mitochondrial function [22,23]. The perspective of the present study was to assess the (patho-) physiological changes associated with hypoxia (0.5% O_2,_ 24 h) induced accumulation of p53 and its translocation to mitochondria in hypertrophied adult human ventricular cardiomyocytes. We also sought to investigate the improvement in efficacy of nanocurcumin in ameliorating hypoxia induced stress in cardiomyocytes compared to curcumin.

In the present study, we found that hypoxia induced hypertrophy in HVCM cells as early as 1 h of hypoxia and reached peak value by 24 h as depicted by increase in ANF levels and FITC-leucine uptake. The early increase in ANF levels depicts that onset of hypertrophy might be an initial adaptive response to hypoxia which further increased with increase in hypoxia exposure. In order to elucidate the molecular pathway by which hypoxia induces cardiomyocytes hypertrophy, we assessed the acetylation status of histones 3 and 4 and simultaneously evaluated the p-300 HAT and HDAC activities. Hypoxia induced hypertrophy was further confirmed by assessing the expression of hypertrophic genes GATA-4 in HVCM cells. It was found that hypoxia (0.5% O_2_, 24 h) stress up-regulated p-300 HAT activity and down-regulated HDAC activity in cardiomyocytes and expression levels of acetylated histones 3 and 4, depicting induction of hypertrophy. These observations are in accordance with previous findings which state that p-300 HAT activities are detrimental in development of myocardial hypertrophy [6,53]. However, for the first time, we provide the experimental proofs that hypoxia stress (0.5% O_2_, 24 h) induces hypertrophy in HVCM cells by up-regulating p-300 HAT and down-regulating HDAC activity. This was confirmed by the observations that phosphorylation and activation of GATA-4 occurred in hypoxia exposed cells. these findings are in accordance with previous studies which state that phosphorylation of GATA-4 occurs in hypertrophied cardiomyocytes under stress [54,55]. Treatment of cardiomyocytes with nanocurcumin significantly down-regulated ANF levels and FITC-phenylalanine uptake depicting down-regulation of hypoxia induced hypertrophy. This was further confirmed by the observation that nanocurcumin treated cells showed significantly down-regulation in acetylation status of histones as depicted by decreased p-300 HAT activity and up-regulation of HDAC activity than curcumin. Also the concomitant observation of restoration of GATA-4 expression in HVCM cells in nanocurcumin treated cells when compared to curcumin confirmed the improvement in therapeutic efficacy of nanocurcumin. Collectively, these observations clearly demonstrate that hypoxia induces hypertrophy in HVCM cells by regulation of p-300 HAT and HDAC activities and GATA-4 levels. Nanocurcumin treatment was found to be highly effective in protecting HVCM cells from hypoxia induced hypertrophy when compared to curcumin.

In order to check whether hypoxia induced hypertrophy was a pathological event, we assessed the mitochondrial function in cardiomyocytes. It was found that disruption in ΔΨ_m_ increased with increase in duration of hypoxia exposure to cardiomyocytes. Hypoxia stress imparted serious oxidative stress to mitochondrial redox machinery and disrupted MnSOD levels within 6 h of exposure. However, these damages were maximized by 24 of hypoxia exposure and were accompanied with caspase-3,-7 activation leading to apoptosis. The parallel decrease ΔΨ_m_ and activation of caspases confirmed that hypoxia induced hypertrophy was indeed a pathological event. These observations suggest that hypoxia (0.5% O_2_) induced hypertrophy might be initially an adaptive cellular strategy (as depicted by increased ANF levels by 1 h of hypoxia) which transforms into pathological form under prolonged stress (24 h). Although cardiomyocyte hypertrophy is an adaptive event to combat increased oxygen demand under hypoxia, but sustained oxygen stress might be lethal to oxygen sensitive cardiomyocytes.

The findings in the present study state that translocation of active p53 to mitochondria was time dependent. It was found that p53 translocated to mitochondria within 1 h of hypoxia and reached maximum by 24 h as depicted by co-immunofluorescence of p53, mitochondrial p53 import-motor protein (mtHsp70 or mortalin) and western blot. Mitochondrial translocation of p53 in cardiomyocytes led to activation of a cascade of events which disturbed mitochondrial homeostasis, cellular redox balance and increased apoptosis. Corroborating to these findings was the observation that there was disruption in ΔΨ_m_ and caspase-3,-7 activation in cardiomyocytes after mitochondrial p53 accumulation. These findings are in accordance with the previous findings of Vaseva *et*. *al*. [56] which state that translocation of p53 to mitochondria by opening mitochondrial permeability transition pore leads to cell death. It is important to note that mitochondrial redox imbalance preceded cytoplasmic redox imbalance, since disturbance in cytoplasmic GSH/GSSG, lipid peroxidation and xanthine oxidase activity was observed only after 6 h of hypoxia exposure. This indicates that localization of p53 disturbs the critical balance of cellular enzymatic and non-enzymatic oxidants. Importantly, we did not find localization of p53 to nucleus indicating that hypoxia (0.5% O_2,_ 24 h) did not trigger nuclear translocation of p53 thus not resulting to DNA-damage in HVCM cells. In order to assess whether hypoxia induced hypertrophy in HVCM cells was dependent translocation of p53 to mitochondria, we assessed the hypertrophy marker ANF by blocking the entry of p53 to mitochondria using cyclosporin A (CsA). It was found that blocking the entry of p53 to mitochondria by CsA did not affect ANF levels in HVCM cells exposed to hypoxia for 24 h. This depicts that induction of hypertrophy was independent of translocation of p53 to mitochondria. These findings are in line with previous reports which state that silencing p53 expression does not prevent cardiomyocyte stress *in vivo* [57]. However, the hypertrophied HVCM cells experienced mitochondrial stress under hypoxia as evident by the data. The data depicts that hypoxia induced hypertrophy appeared as a mal-adaptive response in HVCM cells which disturbed mitochondrial homeostasis due to translocation of p53 and consequently, lead to (patho-)physiological damage in the form of caspase-3,-7 mediated apoptosis.

In order to assess the molecular regulation of translocation of p53 to mitochondria, we assess the expression levels of c-Fos and c-Jun in cardiomyocytes. Recent findings have shown that c-Fos/c-Jun are important negative modulators of p53 and prevent p53 up-regulation mediated cell-cycle arrest or cell-death in a variety of cells [19,58,59]. In the present study, we also found that with increase in duration of hypoxia, enhancement in accumulation of active p53 was associated with down-regulation of c-Fos/c-Jun. Nanocurcumin treatment in cardiomyocytes under hypoxia showed significant up-regulation of c-Fos/c-Jun better than curcumin, depicting improved efficacy in preventing hypoxia induced stress. Also, nanocurcumin was found to be very effective in restoring ΔΨ_m_, restoring MnSOD activity, down-regulating caspase-3,-7 activation and restoring cellular redox status at all the time points when compared to curcumin treated cells under hypoxia. These data confirm the improvement in protective efficacy of nanocurcumin under hypoxia when compared to curcumin.

The cardiomyocytes are imperatively aerobic in nature and consumes large amount of oxygen to sustain normal function. The high oxygen demand of cardiomyocytes is necessary to meet the constant energy expenditure largely by means of generation of ATP by oxidative phosphorylation. Deprivation in oxygen supply may promote de-compensatory and mal-adaptive response which may lead to more severe pathological conditions. Thus, assessment of efficiency in generation of ATP remains important to be assessed under hypoxia. We assessed hypoxia induced changes in mitochondrial function in hypertrophic cardiomyocytes by evaluating bio-energetic efficiency in terms of assessment of ATP generation and p-AMPKα activity as the hallmarks of energy deficit in cells. Increased p-AMPKα activity indicates adaptive response to hypoxia which promotes preservation of ATP for sustaining vital functions and promotes more ATP generation to meet the increased energy demands [60]. In the present study, we found that ATP levels decreased in cardiomyocytes time-dependently in response to increase in duration of hypoxia, along with a corresponding rise in p-AMPKα activity suggesting that prolonged scarcity of oxygen experienced by the hypertrophic cardiomyocytes led to disruption in mitochondrial bio-energetic function and initiated adaptive cellular responses. These findings indicate that early stages of hypoxia induced hypertrophy are certainly associated with energy deficit which led to depletion of cellular ATP pools. The present findings are in line with previous studies which suggest that early stages of microembolism-induced heart failure and cardiomyocyte damage were associated with severe disruption in oxidative phosphorylation and ATP generation, without significant changes in *e*.*t*.*c*. complexes [61]. The maximum disruption of ATP levels and p-AMPKα activity coincided with translocation of p53 to mitochondria and consecutive activation of damaging sequence of events. The co-occurrence of mitochondrial translocation of p53 and decreased p-AMPKα activity indicate that hypoxia induced damaging events in hypertrophied cardiomyocytes might be p-AMPKα activity dependent. These observations are in accordance with previous findings of Jones *et*. *al*. [62]. Also, there was increment in acetyl co-A, pyruvate and lactate concentrations and parallel increase in LDH activity under hypoxia depicting severe metabolic stress.

In order to confirm whether hypoxia induced metabolic shift towards glucose as preferred substrate for generating energy, estimation of glucose uptake levels and western blots of GLUT-1and GLUT-4 were done. Previous studies have reported that foetal isoform of GLUT-1 expression increases in adult myocardium and concomitantly, the adult isoform of GLUT-4 expression levels increase under stress [46,47]. We found that hypoxia stress increased glucose uptake in HVCM cells with corresponding increase in GLUT-1 expression and decrease in GLUT-4 expression levels. This suggests that hypoxia stress induces increment in basal glucose uptake levels by HVCM cells as a substrate for generating more ATP in order to meet the increased energy demand. These findings are in line with previous reports which state that myocardial expression of GLUT-1 increases and GLUT-4 decreases under stress and confirms metabolic shift from lipids to carbohydrates as preferred energy generating substrates as previously reported [51,52]. Our findings hence confirmed that HVCM cells experienced severe oxidative stress and the oxidative metabolism was impaired under hypoxia [63–66]. We also found that nanocurcumin treatment significantly restored acetyl co-A, pyruvate, glucose uptake and lactate concentrations, expression levels of glucose transporters, LDH and p-AMPKα activities along with cellular ATP pools in cardiomyocytes under hypoxia than curcumin depicting improvement in protective efficacy of nanocurcumin compared to curcumin. These data show that nanocurcumin substantially improved mitochondrial bio-energetic function and ensured un-interrupted ATP supply to cardiomyocytes under hypoxia, at least in part by modulating substrate specificity and possibly by regulating the interaction between p-AMPKα and p53 as reported in previous studies [62].

Collectively, the major findings of the present study implicate that hypoxia stress induces hypertrophy in HVCM cells by up-regulating p-300 HAT activity and GATA-4 levels. This was accompanied by accumulation of p53 in mitochondria indicating that, hypoxia induced hypertrophy and associated damages might be dependent upon translocation of p53 to mitochondria. The p53 translocation to mitochondria was c-Fos/c-Jun levels dependent and caused severe damages to mitochondrial metabolic, bio-energetic and redox function along with induction of apoptosis by caspase activation. These cellular damaging events were effectively restored by nanocurcumin treatment in cardiomyocytes when compared to curcumin. The data suggests that hypoxia stress promoted hypertrophy by p-300 HAT and GATA-4 activation induced (patho-) physiological damages by translocation of p53 to mitochondria in HVCM cells. However, whether hypoxia- induced hypertrophy is absolutely dependent upon translocation of p53 to mitochondria remains to be elaborated. Also, nanocurcumin treatment in cardiomyocytes prevented hypertrophy and preserved mitochondrial function and cellular redox homeostasis under hypoxia better than curcumin as depicted by restoration in p-300 HAT, HDAC activities, GATA-4 levels and preventing translocation of p53 to mitochondria. The study provides an insight into usability of nanocurcumin as potential therapeutic agent.

## Conclusion

The present study infers that prolonged hypoxic stress is a causative agent of pathological damages in hypertrophied cardiomyocytes. The data depicts that these pathological damages appear due to translocation of p53 to mitochondria and damages to mitochondrial bioenergetics, metabolic and redox functions. Nanocurcumin treatment protected HVCM cells from hypoxia induced hypertrophy and associated damages better than curcumin, in terms of cellular and mitochondrial bioenergetics and redox function. Also, nanocurcumin treatment prevented switching of preferred energy substrate from lipids to glucose in HVCM cells under hypoxia better than curcumin. The study represents the molecular basis of hypoxia induced cardio-damage and infers that nanocurcumin might be used as a potential therapeutic and cardio-protective agent.

## Supporting Information

S1 Fig Changes in mean fluorescent intensity of p300 HAT in HVCM cells: Figure showing changes in fluorescent intensity of p300 HAT in HVCM cells exposed to hypoxia for 24h. Values are mean ± SD, significant values represented as ^@@^ p≤0.01 *vs* normoxia, *p≤0.05 *vs* hypoxia and ^#^p≤0.01 *vs* hypoxia.
(TIF)

S2 Fig Densitometric analysis: Figure showing densitometric analysis of acetylated histone 3, histone 4, GATA-4 and p-GATA-4 under various experimental groups, normalized to beta actin. Values are mean ± SD, significant values represented as ^@@^ p≤0.01 *vs* normoxia, *p≤0.05 *vs* hypoxia and ^#^p≤0.01 *vs* hypoxia.
(TIF)

S3 Fig Changes in ΔΨ_m_ in HVCM cells under 24 h hypoxia: Figure showing percentage changes in ΔΨ_m_ under various experimental groups exposed to hypoxia for 24h compared to normoxia control. Values are mean ± SD, significant values represented as ^@@^p≤0.01 *vs* normoxia, *p≤0.05 *vs* hypoxia and ^#^p≤0.01 *vs* hypoxia.
(TIF)

S4 Fig Changes in mean fluorescent intensity in MnSOD in HVCM cells: Values are mean ± SD, significant values represented as ^@@^p≤0.01 *vs* normoxia, *p≤0.05 *vs* hypoxia and ^#^p≤0.01 *vs* hypoxia. No significant change was observed in nanocurcumin or curcumin treated cells under normoxia (ns).
(TIF)

S5 Fig Figure showing changes in ΔΨ_m_ under various experimental groups exposed to hypoxia for 24h. Values are mean ± SD, significant values represented as ^@@^p≤0.01 *vs* normoxia, *p≤0.05 *vs* hypoxia and ^#^p≤0.01 *vs* hypoxia. ns depicts non-significant changes.
(TIF)

## Abbreviations

DCFH-DA: Dichlorofluorescein Diacetate
GSH: Glutathione reduced
GSSG: Oxidized Glutathione
h: hours
Hsp: Heat shock protein
MDA: malondialdehyde
MTT: 3-(4,5-dimethylthiazol-2-yl)-2,5-diphenyl-2H-tetrazolium bromide
PBS: Phosphate-Buffered Saline
ROS: Reactive Oxygen Species
